This article has been retracted.

# Comprehensive computational analysis reveals H5N1 influenza virus-encoded miRNAs and host-specific targets associated with antiviral immune responses and protein binding

**DOI:** 10.1371/journal.pone.0263901

**Published:** 2022-05-09

**Authors:** Fatima Noor, Muhammad Hamzah Saleem, Muhammad Rizwan Javed, Jen-Tsung Chen, Usman Ali Ashfaq, Mohammad K. Okla, Mostafa A. Abdel-Maksoud, Yasmeen A. Alwasel, Wahidah H. Al-Qahtani, Huda Alshaya, Ghulam Yasin, Sidra Aslam

**Affiliations:** 1 Department of Bioinformatics and Biotechnology, Government College University, Faisalabad, Pakistan; 2 College of Plant Science and Technology, Huazhong Agricultural University, Wuhan, China; 3 Department of Life Sciences, National University of Kaohsiung, Kaohsiung, Taiwan; 4 Botany and Microbiology Department, College of Science, King Saud University, Riyadh, Saudi Arabia; 5 Department of food sciences & nutrition, College of food & Agriculture sciences, King Saud University, Riyadh, Saudi Arabia; 6 Cell and Molecular Biology, University of Arkansas, Fayetteville, AR, United States of America; 7 Department of Botany, Bahauddin Zakariya University, Multan, Pakistan; Universite d’Orleans, FRANCE

## Abstract

H5N1 virus (H5N1V) is highly contagious among birds and it was first detected in humans in 1997 during a poultry outbreak in Hong Kong. As the mechanism of its pathogenesis inside the host is still lacking, in this *in-silico* study we hypothesized that H5N1V might create miRNAs, which could target the genes associated with host cellular regulatory pathways, thus provide persistent refuge to the virus. Using bioinformatics approaches, several H5N1V produced putative miRNAs as well as the host genes targeted by these miRNAs were found. Functional enrichment analysis of targeted genes revealed their involvement in many biological pathways that facilitate their host pathogenesis. Eventually, the microarray dataset (GSE28166) was analyzed to validate the altered expression level of target genes and found the genes involved in protein binding and adaptive immune responses. This study presents novel miRNAs and their targeted genes, which upon experimental validation could facilitate in developing new therapeutics against H5N1V infection.

## Introduction

Viruses have become a new threat to mankind and thus drawn more attention, because of their potential to cause epidemics [1]. Among which, H5N1V virus (H5N1V) is an avian influenza virus that leads to serious respiratory disorders in birds and is especially deadly for poultry [2]. The transfer of pathogenic virus from poultry to humans ranged an alarming bell for the scientific community to underscore this public threat [3, 4]. The human first case of influenza virus emerged in Hong Kong in 1997, involved 18 patients with 6 deaths [2, 5]. In the last two decades, more than 600 confirmed cases of H5N1V have been recorded in various nation-states [6]. Humans infected with H5N1V represent the symptoms of neurological dysfunction, organ disorders, and acute respiratory distress syndrome (ARDS) [7, 8]. ARDS is the root cause of H5N1V infection mortality. Mostly recognized pathogenesis mechanism for ARDS is host innate immunity dysfunction leading to immoderate chemokines and cytokines release [9, 10]. Various drugs such as Oseltamivir and Zanamivir are being used to treat H5N1 infections. But these drugs has many side effects [11]. However, the actual treatment is yet to discover. Among all influenza viruses, H5N1V has the highest mortality rate [2] that reinforced the attentions of researchers to untangle the intricate molecular mechanism underlying and uncover more enthralling and promising molecular candidates with effective prognostic value.

The H5N1V genome comprises of 8 segments that are encoded by ten proteins named PB2 (length: 759 amino acid(aa)), PB1(length: 757 aa), PA (length: 716 aa), HA (length: 568 aa), NP (length: 498 aa), NA (length: 499 aa), M1(length: 252 aa), M2(length: 97 aa), NS1 (length: 225 aa), and NS2 (length: 121 aa). Supportive care is offered to the affected person for the H5N1V treatment. However, the exact mechanism underlying this viral infection is poorly known. In the era of coronavirus, it has been pointed out that COVID-19 shares symptoms with H5N1V, however, no clear study has been made on it yet. Hence, the bell is ringing slightly, hence its need of the hour to understand the complete mechanisms behind the pathogenesis of H5N1V infection.

Micro-RNAs (miRNAs) are small non-coding RNA molecules [12–14]. In the last half-century, the knowledge regarding miRNAs has become a thirst for researchers [15]. This is just because of the recent advancements in technologies [16]. Bioinformatics approaches and microarray technology enable researchers to identify the potential miRNA involved in the viral infection [17–19]. miRNAs are involved in the post-transcriptional gene expression of countless metabolic pathways through binding with the three prime untranslated regions (3’-UTR) of messenger RNA(mRNA) [20–22]. miRNAs perform their functions by coupling with target mRNA [23, 24]. miRNAs are concerned with the development, proliferation, sustained inflammation, fibrosis, apoptosis, immune response, and so on [25–30]. miRNAs come forward as the targets of interest due to their involvement in metabolic pathways. Multiple studies have shown that miRNAs may have a critical role to play in viral infection [1, 31, 32]. In the past, miRNAs of humans were administered by targeting the associated genes for combating the pathogenesis of infections [33]. Several studies have shown that miRNA is involved in the pathophysiology of Ebola, Zika, and dengue viruses [34]. It’s turning into a great study topic for molecular biology experts all around the globe. More research on miRNAs regarding their contribution to viral infection revealed the potential miRNAs shown to target specific host genes [33, 35].

Numerous studies have been conducted on the H5N1V infection, but currently, there is no sufficient evidence to prove the existence of miRNAs in the H5N1V genome. To tackle this issue, we conducted computational analysis for identifying putative miRNAs in the H5N1V genome. Moreover, the aim of the present study was to find the potential targets of putative miRNAs coupled with their corresponding gene ontologies and KEGG (Kyoto Encyclopedia of Genes and Genomes) pathways. Our findings provide potential H5N1V-produced miRNAs and their targeted genes, which facilitate the pathogenesis and prolonged refuge of the virus in the host. Experimental validation of these miRNAs could facilitate in developing new therapeutics against H5N1V infection.

## Methodology

### Retrieval of H5N1V genome and prediction of pre-miRNA

H5N1V is the most common type of bird flu. Only one strain (A/Goose/Guangdong/1/96) of H5N1V and its genome (accession no. GCF_000864105.1) is available in National Center for Biotechnology Information (NCBI) database, which is a freely accessible public data-hub [36]. Hence, the H5N1V genome (accession no. GCF_000864105.1) was retrieved from NCBI in FASTA format. To predict the presence and positions of the precursor miRNAs (pre-miRNAs) in the genome sequence, we used two ab initio based programs named, VMir (filtered using predefined settings that is, 60 nt set for minimum hairpin size parameter, 220 nt for maximum hairpin size, and 115 minimum for hairpin score) and miRNAFold (https://evryrna.ibisc.univ-evry.fr/miRNAFold) (with a sliding window size of 150 and minimum hairpin size as 0) [37, 38]. miRNAFold is implemented as a web server with an intuitive and user-friendly interface, as well as a standalone version while VMir is provided in a standalone version only. We then used only those precursor miRNAs which were predicted by both of these prediction tools for the purpose of getting high confidence pre-miRNAs only. Stem-loop hairpin secondary structure is one important component to discriminate between pre-miRNA and primary miRNA (pri-miRNAs). The Triplet SVM Classifier tool [39] was utilized to find the true precursor miRNAs among a set of conserved stem-loops. Triplet-SVM classifier can be freely accessible on website; http://bioinfo.au.tsinghua.edu. In the Triplet SVM Classifier tool, the value of the minimum base was set to 22 for the stem-loop.

### Classification of pre-miRNA and validation of secondary structures

To discriminate and validate the real precursor miRNAs from pseudo-pre-miRNAs, we used a Markov model-based tool, FOMmir (https://bioinf.shenwei.me/cgi-bin/FOMmiR.cgi) [40], and an SVM-based tool, iMiRNA-SSF(http://bliulab.net/iMiRNA-SSF/) [41] with their default parameters. Furthermore, we examined the stable secondary structure within these real pre-miRNAs by RNAstructure webserver (https://rna.urmc.rochester.edu/RNAstructureWeb/) [42]. Finally, only those pre-miRNAs were retained which satisfy all these filtering criteria to minimize the chances of false-negative results.

### Identification of mature miRNAs

With the purpose of extracting the mature miRNA position from the pre-miRNA hairpins, matureBayes (http://mirna.imbb.forth.gr/MatureBayes.html) [43], MiRduplexSVM [44] were used. MiRduplexSVM is freely available for use as a web-service at http://139.91.171.154/duplexsvm/. These tools use SVM based model for distinguishing the mature miRNAs and also provide information regarding the strand of mature miRNAs.

### Prediction of host specific target gene

miRNA exert their effect by targeting three prime untranslated regions (3’-UTR) of messenger RNA (mRNA). Host-pathogen interactions are vital to our understanding of the infectious disease. Therefore, the prediction of the target gene might assist in understanding the disease pathogenesis in the host. First of all, we retrieved 3’-UTR sequences of the homo sapiens protein-coding genes from the Ensembl biomart(https://www.ensembl.org/biomart/index.html) [45].

Then, RNAhybrid (https://bibiserv.cebitec.uni-bielefeld.de/rnahybrid) (with default parameters and cutoff of ((probability value))p-value < 0.05 to filter target genes) [46], psRNATarget (http://plantgrn.noble.org/psRNATarget/) (Expectation ≤ 3, a slightly relaxed threshold) [47], and IntaRNA 2.0 (http://rna.informatik.uni-freiburg.de/IntaRNA) (with parameters–model = X,–outMode = C,–mode = H, mfe ≤ − 10 kcal/mol,) [48] were employed in order to identify the host-specific target genes of predicted miRNAs. Only those targets were retained which were predicted by at least two prediction tools in order to obtain high confidence targets only.

### Functional enrichment analysis of targeted genes

Pantherdb (http://www.pantherdb.org/) and KEGG (https://www.genome.jp/kegg/) database were utilized to perform functional enrichment analysis and pathway analysis respectively [49, 50]. The target genes were subjected to Pantherdb to find the enriched gene ontology and pathways involving the microRNA target genes. P-values for multiple testing was adjusted using Hochberg’s method of False Discovery Rate (FDR) [51] and a cut-off of FDR<0.05 was utilized.

### Analysis of gene expression profile

Gene Expression Omnibus (GEO) (https://www.ncbi.nlm.nih.gov/geo/) [52] is a freely available public repository of the National Center for Biotechnology Information (NCBI), which encloses the gene profiles. The expression level of each target gene was obtained from the microarray dataset GSE28166. This expression dataset was based on the GPL6480 platform (Agilent-014850 Whole Human Genome Microarray 4x44K G4112F), which contained 36 samples, including 18 controls samples and 18 H5N1V-infected samples. Limma R package [53] was used to find out significant differentially expressed genes (DEGs) from this study. For this study, we used uninfected cells (GSM697564, GSM697565, GSM697566) as control and perform the analysis twice, one for the replicates of 12-hours H5N1V-infected samples (GSM697591, GSM697592, GSM697593) and another is for 24-h H5N1V-infected samples (GSM697597, GSM697598, GSM697599). Processing the data indicated the Log2 fold changes in total human genes’ expression level and target genes expression level were analyzed at the same time by setting the significance levels at adj. p-value < 0.05). Only those genes are to be significantly expressed genes that have logFC value ±1 with adjusted p-value <0.05. If the logFC value is negative then that gene is marked as downregulated and the gene having the logFC value in positive is called upregulated. Another round of functional enrichment analysis was performed for the downregulated target genes of the predicted miRNAs using the Pantherdb and KEGG database. Moreover, the overall methodology that is used for the prediction of miRNA along with their target genes is outlined in **Fig 1.**

**Fig 1:** Graphical synopsis of representing the overall strategy used in the prediction of miRNA and their cellular targets.

## Results

### Retrieval of H5N1V genome and prediction of real pre-miRNAs

To identify whether H5N1V produces any miRNAs, we utilized two ab initio based tools; Only 20 putative pre-miRNAs were generated by Vmir, while 150 were generated by miRNAFold. Among all these predicted pre-miRNAs, we took only 14 pre-miRNAs which were predicted by Vmir and miRNAFold for the purpose of getting high confidence pre-miRNAs only. We considered these 14 pre-miRNAs for further analyses. Hence, by this way, we obtained 14 pre-miRNAs with the length varies between 67–139 nucleotides (Table 1). All pre-miRNAs are predicted to be truly positive by Triplet SVM Classifier. We further refine the sequences of true pre-miRNAs through iMiRNA-SSF and FOMmir and obtained a set of 9 real pre-miRNAs, from which either one or both strands can form a functional miRNA (mature miRNA). From these 9 pre-miRNAs, 5 were present on reverse orientation whereas the rest of the 4 miRNAs were present on direct orientation. Furthermore, we validate the minimum free‐energy (MFE) value of pre-miRNA sequences using RNAstructure webserver (Fig 2). The MFE value for every pre-miRNA was calculated and values ranged from -17.0 kcal/mol, to -46.3 kcal/mol having a mean of -30 kcal/mol. MFE values along with the positional entropy of 9 real pre-miRNAs are present in Table 1.

**Fig 2:** Minimum free‐energy (MFE) value in RNAstructure webserver and the MFE secondary structure and positional entropy of 9 real pre-miRNAs were created. (A) MD96; (B) MR124; (C) MR46; (D) MD105; (E) MD76 (F)MR90 (G) MD94 (H) MR64 (I) MD101.

**Table 1:** pre-miRNA obtained from VMir and further validated using imiCRNA and RNAstructure.

Sr.no#	miRNA name	Orientation	Sequence	Genome location	Size, nt	MFE, kcal/mol
1	H5N1V-MD96	Reverse	GGCAGCGGAAGCCATGGAGGTTGCTAGTCAGGCTAGGCAGATGGTGCAGGCAATGAGGACAATTGGGACTCATCCTAGCTCCAGTGCCGGTCTGAAAGATAATCTTCTTGAAAATTTGCAGGCC	12576–12699	124	-46.3
2	H5N1V-MR124	Reverse	AGTGGGTTGGTGGTAGTTGCCATCTGTCTGTGAGACCGATGCTGTGAATCTGCAATCTGCTCACAAGTGGCACACACTAGGCCAAAAGCCACT	12405–12497	93	-30.7
3	H5N1V-MR46	Reverse	TGGGTATCTGTAGTCCTTAATGAATAGCTGAAGAGCCATCTGAGCTGTTGCTGGTCCAAGGTCGTTGTCCATCATATTGTTCTTTATCACTGTAACACCAATGCTCATGTCAGCCGATTCATTAATCCCAGACACTCCA	3948–4086	139	-33.8
4	H5N1V-MD105	Direct	AGATGGCTCATTGCTGAATGTAGAAATATACTGACAAAGACTGAAAATAGCTTTGAACAGATAACATTTTTGCAAGCATTGCAACTCT	13735–13822	84	-17.0
5	H5N1V-MD76	Direct	TCGTGCCTTCCTTTGACATGAGTAATGAAGGATCTTATTTCTTCGGAGACAATGCAGAGGAATATGA	10342–10390	67	-20.7
6	H5N1V-MR90	Reverse	TAGCATTCTGGCGTTCTCCACCAGTTTCCATCTGTTCATAAGATCGTTTGGTGCCCTGAGACGCCATGATGTTG	8894–8967	74	-26.6
7	H5N1V-MD94	Direct	AGTGGCTTTTGGCCTAGTGTGTGCCACTTGTGAGCAGATTGCAGATTCACAGCATCGGTCTCACAGACAGATGGCAACTACCACCAACCCACT	12405–12497	93	-28.5
8	H5N1V-MR64	Reverse	GGATCCAGCTTGCTAGTGATCTAGGCTTTGGTTCATCACTGTCATACTGCCTTAGATCGCTAACATCTTTGCAATCC	5946–6022	77	-21.4
9	H5N1V-MD101	Direct	AGCTACTCAGTATGAGAGACATGTGTGATGCCCCCTTTGATGACAGGCTCCGAAGAGACCAAAAGGCATTAAAGGGAAGAGGCAGCACACTTGGACTCGATTTAAGAGTGGCT	13093–13205	113	-45.6

### Identification of mature miRNAs

We found the position and sequence of 18 mature miRNAs within the validated precursor miRNA sequences utilizing the matureBayes and MiRduplexSVM tools. Either one or both of the strands in a real pre-miRNA sequence can perform the function of mature miRNA. Out of these 18 mature miRNAs, 9 mature miRNAs were present on 5′arm of the stem of the potential hairpin loop structure while 9 were present on 3′arm of stem-loop hairpin structure (**Table 2**).

**Table 2:** Length, location and predicted miRNAs sequence of RSN mature miRNAs.

Sr.no#	miRNA name	Location	Length of mature miRNAs	Predicted miRNA sequence
1	H5N1V-MD96	5	23	UAGGCAGAUGGUGCAGGCAAUGA
2	H5N1V-MD96	3	21	CUAGCUCCAGUGCCGGUCUGA
3	H5N1V-MR124	5	23	UUGCCAUCUGUCUGUGAGACCGA
4	H5N1V-MR124	3	22	AAUCUGCUCACAAGUGGCACAC
5	H5N1V-MR46	5	22	UAGCUGAAGAGCCAUCUGAGCU
6	H5N1V-MR46	3	21	CAAUGCUCAUGUCAGCCGAUU
7	H5N1V-MD105	5	22	UGAAUGUAGAAAUAUACUGACA
8	H5N1V-MD105	3	23	UGAACAGAUAACAUUUUUGCAAG
9	H5N1V-MD76	5	22	UCCUUUGACAUGAGUAAUGAAG
10	H5N1V-MD76	3	21	UCGGAGACAAUGCAGAGGAAU
11	H5N1V-MR90	5	22	UGGCGUUCUCCACCAGUUUCCA
12	H5N1V-MR90	3	22	UUUGGUGCCCUGAGACGCCAUG
13	H5N1V-MD94	5	19	UGCCACUUGUGAGCAGAUU
14	H5N1V-MD94	3	22	UCGGUCUCACAGACAGAUGGCA
15	H5N1V-MR64	5	21	UUGCUAGUGAUCUAGGCUUUG
16	H5N1V-MR64	3	22	UACUGCCUUAGAUCGCUAACAU
17	H5N1V-MD101	5	23	UGAGAGACAUGUGUGAUGCCCCC
18	H5N1V-MD101	3	22	AGGCAGCACACUUGGACUCGAU

### Prediction of gene targets for putative H5N1V miRNAs

After finding the functional mature miRNAs, we employed 3 different miRNA-target prediction software, the psRNATarget tool predicts 70 gene targets while RNAhybrid and IntaRNA predicted 35 and 55 genes, respectively. Among all these predicted genes, we picked only 41 genes for further analysis which were predicted by at least two of the gene targets prediction tools. Furthermore, out of these 41 targeted genes, only 35 genes were found as significant targets as they showed adjusted p-value(probability value) < 0.05 (**S1 Table in S1 File**). Previously, miRNAs produced by RNA viruses such as HIV-1, Dengue virus, West Nile virus, and Ebola virus were reported and all these followed the same strategy for prediction of gene targets from viral miRNAs [34]. Following that, viral miRNAs predicted in this study might target the genes which facilitate their own replication, transcription, and/or translation and consequently help the virus to hijack these pathways for the successful completion of its life cycle.

### Functional enrichment analysis

We performed functional enrichment analysis by pantherdb and KEGG database, to better understand the functional significance of targeted genes produced by the putative miRNAs of H5N1V. These tools revealed functionally enriched pathways and biological processes associated with DNA binding, protein binding, cMAP signaling, signaling pathways, signal transduction, and metabolic pathways. Table 3 enlists the targeted genes along with their associated pathways.

**Table 3:** Functional analysis of targeted genes.

Gene name	Gene name	Molecular function	Biological Processes	Cellular components	KEGG
ZYG11B	Protein zyg-11 homolog B	Protein binding	Protein quality control for misfolded or incompletely synthesized proteins, positive regulation of proteasomal ubiquitin-dependent protein catabolic process	Cul2-RING ubiquitin ligase complex	_
ZNF579		DNA binding, RNA binding, metal ion binding	_	Nucleus	_
LASP1	LIM and SH3 domain protein 1	Actin filament binding, protein binding, metal ion binding, cadherin binding, ion transmembrane transporter activity	Ion transport, ion transmembrane transport	Focal adhesion, cytoplasm, cortical actin cytoskeleton	_
RAPGEF3	Rap guanine nucleotide exchange factor 3	Protein domain specific binding, protein binding, guanyl-nucleotide exchange factor activity, cAMP binding	Signal transduction, small GTPase mediated signal transduction, adaptive immune response, positive regulation of GTPase activity, regulation of catalytic activity, cellular response to cAMP, Rap protein signal transduction, regulation of actin cytoskeleton reorganization, and cAMP-mediated signaling	extracellular exosome, microvillus, membrane, endomembrane system, filopodium, plasma membrane, cortical actin cytoskeleton, lamellipodium	Rap1 signaling pathway, cAMP signaling pathway, phospholipase D signaling pathway,adrenergic signaling in cardiomyocytes, leukocyte transendothelial migration, long-term potentiation, serotonergic synapse
FADS2	Acyl-CoA 6-desaturase	Stearoyl-CoA 9-desaturase activity, protein binding, linoleoyl-CoA desaturase activity	unsaturated fatty acid biosynthetic process, lipid metabolic process, linoleic acid metabolic process, alpha-linolenic acid metabolic process	endoplasmic reticulum membrane, integral component of plasma membrane, membrane, integral component of membrane	Alpha-Linolenic acid metabolism, biosynthesis of unsaturated fatty acids, metabolic pathways, fatty acid metabolism, PPAR signaling pathway
SLC4A11	Sodium bicarbonate transporter-like protein 11	Anion antiporter activity, transmembrane transporter activity, proton channel activity, sodium channel activity, symporter activity, protein dimerization activity, inorganic anion exchanger activity, active borate transmembrane transporter activity, bicarbonate transmembrane transporter activity	Inorganic anion transport, sodium ion transport, transmembrane transport, fluid transport, proton transmembrane transport, sodium ion transmembrane transport, ion homeostasis, bicarbonate transport, cellular cation homeostasis, borate transmembrane transport, borate transport	Vesicle membrane, membrane, integral component of membrane, basolateral plasma membrane, plasma membrane, apical plasma membrane	_
ABCA7	Phospholipid-transporting ATPase ABCA7	ATPase activity, ATP binding, ATPase-coupled transmembrane transporter activity, phospholipid transporter activity, phosphatidylserine floppase activity, lipid transporter activity, apolipoprotein A-I receptor activity, phosphatidylcholine floppase activity, floppase activity	Plasma membrane raft organization, negative regulation of endocytosis, negative regulation of MAPK cascade, negative regulation of amyloid-beta formation, regulation of amyloid precursor protein catabolic process, visual learning, positive regulation of phospholipid efflux, memory, phospholipid translocation, amyloid-beta clearance by cellular catabolic process, positive regulation of cholesterol efflux, protein localization to nucleus, amyloid-beta formation, high-density lipoprotein particle assembly, apolipoprotein A-I-mediated signaling pathway, transmembrane transport, positive regulation of protein localization to cell surface, positive regulation of engulfment of apoptotic cell, positive regulation of amyloid-beta clearance, negative regulation of PERK-mediated unfolded protein response, negative regulation of amyloid precursor protein biosynthetic process, lipid transport, positive regulation of ERK1 and ERK2 cascade, phagocytosis, cholesterol efflux, peptide cross-linking, regulation of lipid metabolic process, positive regulation of phagocytosis, phospholipid efflux	Early endosome membrane, glial cell projection, intracellular membrane-bounded organelle, integral component of membrane, cell junction, ruffle membrane, Golgi membrane, endoplasmic reticulum, Golgi apparatus, phagocytic cup, plasma membrane, cell surface	ABC transporters
DEDD2	DNA-binding death effector domain-containing protein 2	DNA binding, protein binding, signaling receptor complex adaptor activity	Cellular homeostasis, negative regulation of transcription, DNA-templated, apoptotic nuclear changes, apoptotic process, rRNA catabolic process, RNA processing, regulation of apoptotic process, positive regulation of extrinsic apoptotic signaling pathway, extrinsic apoptotic signaling pathway via death domain receptors, intracellular signal transduction	Nucleolus, nucleoplasm	_

### Gene expression microarray analysis

To examine the differential gene expression level of putative targets, we utilized the microarray dataset GSE28166 of H5N1V infected Calu-3 cells. LogFC values of gene expression were computed by comparing the control samples to H5N1V infected samples. A total of 1,000,000 genes were discovered by profiling the infected cell for 12hours, from which 170 were down-regulated and 110 were up-regulated, while 20,000 genes were discovered to be unregulated by profiling the infected cells for 24hours (150 were down-regulated and 90 were up-regulated). The comparison among targeted genes with these unregulated genes led to the discovery of 8 genes that were found to be unregulated in both 12 hours and 24 hours infection samples.

Furthermore, we tried to explain the function enrichment analysis of significant targeted genes of the putative miRNAs. In this regard, one more ride of the functional annotation was performed using 8 significant targets and we found that these significant genes are involved in Rap1 (Ras-proximate-1) signaling pathway, in protein binding, adaptive immune responses, PPAR (Peroxisome Proliferator-Activated Receptors) signaling pathway, signal transduction, cAMP signaling pathway, and RNA processing. Later, Funrich tool was used to explore the interaction among eight significant genes and their related neighboring genes. The interaction of eight genes and their related genes was then visualized in form of interaction network (**Fig 3**).

**Fig 3:** The PPI network of the eight genes, and their related genes, created by the FunRich software. Red nodes represents eight significant genes filtered through gene expression analysis, while green nodes represents neighboring genes of the eight genes.

## Discussion

Avian influenza viruses naturally circulate in wild aquatic birds but are easily transmitted to poultry. Occasionally, they can infect humans who come into close contact with infected birds, for instance at wild poultry markets or commercial farms [10, 54, 55]. H5N1V is considered the leading cause of acute respiratory distress syndrome [56]. During the poultry outbreak in 1997 outbreaks, 18 farmers were infected with the H5N1V virus. Of these 18 infected people, 6 people died as the death rate is higher than 60% [57]. In the early years, multiple mechanisms involved in H5N1V pathogenesis is poorly known [58]. Our functional annotation of host-specific target genes by H5N1V’s miRNAs might be helpful in understanding this targeted slicing on the pathogenesis of H5N1V. Finally, validation of targeted genes was performed through the microarray dataset (GSE28166). Validation of genes with differential expressed genes (DEGs) of infected H5N1V patients has led to the identification of eight significant genes named ZYG11B, ZNF579, LASP1, RAPGEF3, FADS2, SLC4A11, ABCA7, and DEDD2.

Viruses retain multiple constantly evolving policies to subvert the host cellular environment. The interaction among the cell-cycle machinery of the host with the protein of virus is not necessarily favorable for the life cycle of the host [59] (Fan et al., 2018). However, in the case of H5N1V, there is no study available regarding the H5N1V’s interruptions in these processes. In the current analysis, we discovered many target proteins that are found to participate in metabolic pathways, PPAR signaling pathway, Rap1 signaling pathway, cAMP signaling pathway, serotonergic synapse, and phospholipase D signaling pathway of the host. These whole processes reveal the capability of H5N1V miRNAs for exerting great control over the host-cellular machinery.

Thousands of RNA viruses spread contagious diseases in animals. The single-stranded nature of viral genomes draws more attention of the researchers to utilize several RNA binding proteins of virus and host to better understand the underlying mechanisms behind the pathogenesis [60]. By considering the current analysis majority of proteins namely ZYG11B, LASP1, FADS2, DEDD2, and RAPGEF3 discovered to participate in protein binding.

The immune response is activated by the identification of a conserved pattern in the associated antigenic structure of viruses [61]. There is a dynamic change in the immune response in the host body during the infection of viruses [62]. According to our findings, RAPGEF3 participated in the adaptive immune response of the host. These findings conclude that the miRNAs of H5N1V targeted the genes that interfere with the immune responses in the host, which unfortunately lead to H5N1V infection in humans.

It is also noteworthy that target genes named RAPGEF3 and DEDD2 are associated with pathways concerned with the signal transduction in the host. Recently, it has been investigated that H5N1V directly infected the cellular signaling events hence inhibit the activation of signal transduction pathways. These signal transduction pathways are aimed to protect humans against H5N1V. This inhibition leads to the impairment in the signal transduction pathways in the host. Following that, it gives clear evidence that H5N1V’s miRNAs directly target the RAPGEF3 and DEDD2 in humans which causes disruption in signal transduction pathways. As in the case of HIV, the HIV cAMP signaling pathway contribute to T cell dysfunction which in turn causes impairment and reduces cytokines production. Our analysis proposed that RAPGEF3 are involved in the cAMP signaling pathways which infer that the miRNAs of H5N1V targeted these genes interfere with the cAMP signaling pathways in the host and caused H5N1V infection in humans.

Viruses caused disruption in the cellular homeostasis of the host which may turn off the luxury function of the cell. This disrupts cellular homeostasis and causes infection. Our findings proposed that DEDD2 participated in the cellular homeostasis, hence these host genes were found to be targeted by the H5N’s miRNAs associated with the cellular homeostasis. Majority of the viral infection leads to the cell death in the host. Considering our analysis, DEDD2 was discovered to be associated with the apoptotic signaling pathway, hence these host genes were found to be targeted by the H5N1V’s miRNAs concerned with apoptosis. miRNAs carry out their functions by coupling with a target mRNA [63]. Proteins named DEDD2 are discovered to be directly involved in RNA processing.

More importantly, HIV-1, West Nile virus, Ebola virus, and mosquito-borne Dengue virus has also been reported to encode miRNA like small viral RNAs [32]. In this context, we hypothesize that H5N1V-encoded miRNAs modulate host immune system and various physiological functions that provide the viruses selective advantages for prolonged refuge and disease pathogenesis within the host. Moreover, Hong et al. an [64] and Li et al. [4] predicted various H5N1V encoded miRNAs. However, no study has reported miRNAs produced by H5N1V target genes after analyzing the complete genome. Hence, this study will pave the way for future research. Since the present study is based on an integrated computation pipeline, thus requires additional laboratory tests.

These findings validate the present conclusion that the miRNAs of H5N1V might target the host-specific gene. With reference to our findings, we introduce a new mechanism underlying the pathogenesis of H5N1V by means of miRNA-mediated gene silencing.

## Conclusion

In this study, we propose a mechanism, which portrays that H5N1V may progress its pathogenesis through producing miRNA that targets the genes involved in multiple pathways in the host. Some of these pathways include protein binding, cMAP signaling pathways, adaptive immune responses, apoptotic signaling pathways, signal transduction, and metabolic pathways. Our research will serve as a significant pioneer for the researchers who want to identify the associated pathways involved in the pathogenesis of H5N1V. Additional experimental research (such as quantitative reverse transcription polymerase chain reaction, miRNA microarray, and RNA sequencing) on these putative miRNAs leads to an increase in our knowledge to fight against H5N1V in the future by means of novel therapeutic approaches.

## Supporting information

S1 File (DOCX)
